# Machine Learning-Based MRI LAVA Dynamic Enhanced Scanning for the Diagnosis of Hilar Lesions

**DOI:** 10.1155/2022/9592970

**Published:** 2022-02-24

**Authors:** Haijin Wang, Song Wang, Lihua Zhou

**Affiliations:** ^1^School of Nursing, Anhui Medical University, Hefei, China 230032; ^2^Department of Hepatobiliary and Pancreatic Surgery, The First Affiliated Hospital of Anhui Medical University, Hefei, China 230022; ^3^Medical imaging center, The Fourth Affiliated Hospital of Anhui Medical University, Hefei, China 230002

## Abstract

**Objective:**

To explore the value of machine learning-based magnetic resonance imaging (MRI) liver acceleration volume acquisition (LAVA) dynamic enhanced scanning for diagnosing hilar lesions.

**Methods:**

A total of 90 patients with hilar lesions and 130 patients without hilar lesions who underwent multiphase dynamic enhanced MRI LAVA were retrospectively selected as the study subjects. The 10-fold crossover method was used to establish the data set, 7/10 (154 cases) data were used to establish the training set, and 3/10 (66 cases) data were used to establish the validation set to verify the model. The region of interest was extracted from MRI images using radiomics, and the hilar lesion model was constructed based on a convolutional neural network.

**Results:**

There were significant differences in respiration and pulse frequency between patients with hilar lesions and without hilar lesions (*P* <0.05). The subjective scores of the images in the first three phases of dynamic enhanced scanning in the training set were higher than those in the validation set (*P* < 0.05). There was no significant difference between the training and validation set in the last three phases of dynamic enhanced scanning.

**Conclusion:**

Machine learn-based MRI LAVA dynamic enhanced scanning for diagnosing hilar lesions has high diagnostic efficiency and can be used as an auxiliary diagnostic method.

## 1. Introduction

Magnetic resonance imaging (MRI) has been widely used in clinical diagnosis because of its safety, no radiation, high soft tissue resolution, multidirectional, and multiparameter [1]. The anatomical structure of the hilar region is complex, and the incidence rate is high. Therefore, MRI has irreplaceable advantages as an essential method to check hilar lesions [2]. Liver acceleration volume acquisition (LAVA), as a new MRI imaging technology with high time resolution, can obtain images at different times. The dynamic enhancement features of lesions can be displayed in more frequent sequences, often used in dynamic enhancement imaging. However, this sequence is greatly influenced by the patients' respiratory movement, which largely determines the quality of MRI [3].

Hilar lesions need to consider the anatomical location, scope, and relationship with peripheral blood vessels of the tumor [4]. Therefore, it is essential to obtain clear and high-quality images of hilar hepatic without artifacts. Radiomics is a noninvasive method for identifying quantitative imaging indicators to predict critical clinical outcomes [5, 6]. This technology combines imaging and machine learning to extract high-throughput quantitative features from clinical images [7]. In recent years, studies have shown that convolutional neural network (CNN) machine learning based on deep learning architecture can automatically perform image classification by providing supervised input-output data [8–11]. However, there are few reports about applying this model in the imaging examination of hilar lesions.

The purpose of this study was to explore the value of machine learning-based MRI LAVA dynamic enhanced scanning for the diagnosis of hilar lesions to provide clinicians with an auxiliary diagnostic method for hilar lesions.

## 2. Materials and Methods

### 2.1. General Information

A random sampling method was used to select 90 patients with hilar lesions clinically found from July 2019 to October 2019 who underwent multiphase dynamic enhanced MRI LAVA examination. In addition, 130 patients without hilar lesions who underwent this examination were selected.

Inclusion criteria are as follows: (1) Patients had no contraindications for MRI examination, and all underwent multiphase LAVA dynamic enhanced scanning for the first time. (2) Patients can cooperate with examination, with no mental diseases. (3) Before the examination, all patients were truthfully informed about the content of this study, obtained and signed informed consent.

Exclusion criteria are as follows: (1) patients allergic to contrast agents; (2) patients with underlying severe diseases; (3) patients with vague mental consciousness and lack of cognitive ability; and (4) patients having a cardiac pacemaker or metal implant.

A 10-fold crossover method was used to establish a data set for all 220 patients. 7/10 data (*n* = 154 cases) established a training set, including 82 males and 72 females, aged 19-81 years, with an average of (51.5 ± 14.9) years. A validation set was established in 3/10 data (*n* = 66 cases), including 36 males and 30 females, aged 18-81 years, with an average of (52.0 ± 16.6) years. Then, the machine learning model was constructed, and its performance was evaluated. The modeling flow chart is shown in Figure 1.

### 2.2. Scanning Method

The images were obtained in the GE Signa HDx 3.0 T MRI system, body phased-array surface coil. The scanning sequence included axial T1WI, axial iso phase inversion, coronal T2WI, axial fat compression T2WI, DWI (*b* = 800 s/mm^2^), magnetic resonance cholangiography (MRCP), and LAVA multiphase dynamic enhancement sequence. The scanning process is as follows: After plain scanning, 0.1 mmol/kg (gadolinium spray meglumine, GD-DTPA) was injected through the cubital vein mass at a flow rate of 2.0 mL/s, followed by injection of 20 mL normal saline, and dynamic scanning was performed in six phases (phase A1-A6). 10 s after the contrast agent injection, the patients were instructed to hold their breath for about 15-20 s for stage A1 scan. After each scan, patients were instructed to take a deep breath, followed by stage a2-a5 scan at 55, 90, 120, 180, 240, and 360 s. The holding time for each phase was 15-20 s.

### 2.3. MRI Interception

After preprocessing the experimental images, the image was segmented into regions of interest (ROI). The tumor was separated from other tissues by a circle corresponding to the size of the hilar tumor to calibrate the tumor region. The ROI images were collected using radiomics **(**Figure 2**)**.

### 2.4. Data Collection

Typical CNN consists of a convolution layer and pooling layer. The basic structure of the convolutional neural network is shown in Figure 3. The convolution layer can directly conduct convolution operations with two-dimensional data, read images, and identify their features. As the core of CNN, the convolution layer is used to extract the features of input data. The convolution layer extracts local information from the data sampled regularly, and each convolution layer is composed of multiple filters. After the convolution, an activation graph describing the existing degree of features in the data is generated [12]. In general, the output of the JTH filter in the one-dimensional convolution layer is

(1) $$\begin{array}{c} x_{j}^{l}=\text{ReLU}\left(\underset{i\in D}{\sum }x_{i}^{l-1}*w_{ij}^{l}+b_{j}^{l}\right) \end{array}$$

In machine learning, regularization is used to train set observations to prevent overfitting. For the cost function *J*(*θ*; *X*, *y*), with grid parameter *θ*, the function corresponding to the *J*-th layer of the training set is

(2) $$\begin{array}{c} \hat{J}\left(\theta ;x,y\right)=J\left(\theta ;x,y\right)+\lambda_{1}{\left\|w\right\|}_{1}+{\left\|w\right\|}_{2}. \end{array}$$

### 2.5. Evaluation Index

The image quality of the training set and validation set was graded by two attending physicians. The dynamic enhanced scan's six-phase images (phases A1-A6) were evaluated separately as follows: 1 point: the image was clear and without any motion artifact; 2 points: the image is clear, with a few motion artifacts; 3 points: there are certain motion artifacts, the image is still clear, the lesions can be displayed, and their enhancement features are not affected; 4 points: the motion artifact was obvious, the image was not clear, and the lesion could be displayed to a certain extent, but it had a great influence on the diagnosis; 5 points: the motion artifact was significant, the image was not clear, and could not be used for diagnosis.

### 2.6. Statistical Analysis

SPSS 20.0 statistical software was used to analyze and process relevant data. Independent sample *t*-test was used for measurement data comparison, and an independent sample nonparametric statistical Mann–Whitney rank-sum test was used for image scoring. *P* < 0.05 was considered statistically significant.

## 3. Results

### 3.1. General Conditions

There were no significant differences between the training set and the validation set in gender, age, and proportion of hilar lesions (*P* > 0.05), as shown in Figure 4. There were significant differences in respiration and pulse frequency between these two sets (*P* < 0.05, Table 1).

### 3.2. Image Quality Score

Patients with good breath-holding coordination during dynamic enhanced scan showed clear, dynamic enhancement characteristics of hilar lesions and liver parenchyma, which could meet the diagnostic requirements **(**Figure 5**)**. For patients with poor breath-holding coordination, the image artifacts were heavier or even completely deformed, which could not meet the diagnostic needs **(**Figure 6**)**. The image data in the training set were integrated into the CNN model to obtain the scoring results of important features **(**Table 2**)**. The number of image cases with 1 score and the image quality in first three stages (A1-A3) was statistically significant (*P* < 0.05). The number of image cases and the image quality in last three stages (A4-A6) were not statistically significant (*P* > 0.05).

## 4. Discussion

Hilar lesions are a widespread disease, especially cholangiocarcinoma [13]. At present, dynamic enhanced sequence MRI LAVA is the best imaging method for diagnosing and differential hilar lesions [14]. By obtaining dynamic enhanced multiphase images, more accurate information about blood perfusion of hilar lesions can be provided. Since most patients have different degrees of anxiety, anxiety inferiority complex, and other corresponding negative emotions, a 3.0 T MRI abdominal scan is performed in a dark and closed environment. In addition, patients must be coordinated with regular breath and breath-holding during the dynamic enhanced scan, and the whole examination process takes a long time and is difficult to coordinate. These negative emotions will affect the coordination degree of patients' examination and the accuracy of scanning site structure image and lead to various uncomfortable symptoms such as dizziness, palpitation, and nausea. Eventually, the diagnosis and treatment effect is not good [15]. Therefore, there is still a specific risk of misdiagnosis in the traditional diagnostic methods.

Radiomics based on machine learning can build models according to the information provided by the training sets and then predict the input sample information. In recent years, radiomics has been widely used in diagnosing brain dysfunction and lung cancer by MRI [16, 17]. Combining radiomics with disease imaging can mine the underlying information of related images, which can be applied to individual diagnosis and prognosis assessment [18]. This study showed that the respiratory and pulse scores of patients in the training group with hilar lesions were lower than those in the without hilar lesions group (*P* < 0.05), which indicates that the machine learning model has better prediction reliability and is effective in improving diagnostic efficiency. Our results are similar to previous studies [19]. Liu et al. assisted in the preoperative classification of HCC based on MRI radiomics. They found that the radiomics model based on unsupervised learning descent mode had a good predictive performance in the identification of pathological classification [20]. Zhang et al. established a model based on machine learning to intercept the region of interest of primary liver cancer tumors in CT images. Their results showed that the features of high-throughput images could be effectively extracted, and the prediction model had good identification efficiency in different pathological types [21].

As one of the essential factors for the success of MRI LAVA dynamic enhancement, respiratory coordination determines the length of examination to a certain extent and determines the quality of diagnostic images [22]. However, in a convolutional neural network based on deep learning architecture, many high-dimensional and quantitative image features are extracted from MRI images at high throughput for analysis [23, 24]. The results show that the image quality of the training set is better than that of the verification set in the first three phases (A1-A3 phase), which indicates that the model can effectively extract practical features, verify the validity of the model, and improve the image quality. The image quality of the last three phases (A4-A6) did not improve. The possible reasons are analyzed as follows: (1) Due to the experimental scanning method of end-expiratory breath-holding, patients are more prone to involuntary movement in the late stage of breath-holding with the extension of breath-holding time. In addition, the total time of the six dynamic scans was longer than that of the available scans, which would significantly increase the possibility of motion artifacts in the later stage of breath-holding. (2) The imaging time of each phase of the LAVA dynamic enhancement scan sequence is shorter, so the influence of patients' respiratory movement on the LAVA dynamic enhancement sequence is more significant than that of the conventional sequence. In general, machine learning-based MRI LAVA dynamic enhanced scanning has good predictive efficacy in MRI diagnosis of hilar lesions.

There are some limitations to our study. Machine learning needs to extract feature parameters from images during classification and recognition and then carry out targeted analysis, which may miss some critical information and reduce the model's accuracy [25, 26]. In addition, the sample of this study was a single-center retrospective study, which needs further verification in the prospective study of a large multicenter sample.

## 5. Conclusion

In conclusion, machine learning-based MRI LAVA dynamic enhanced scanning in this study has stable and reliable results of LAVA dynamic enhancement examination for patients with hilar lesions. The imaging quality has been improved, providing an auxiliary means for clinicians to diagnose.

## Figures and Tables

**Figure 1:** Modeling flow chart.

**Figure 2:** Capture of hilar region of interest for MRI.

**Figure 3:** Schematic diagram of convolutional neural network.

**Figure 4:** General data comparison of patients in training and test sets. There were no significant differences in gender (a), proportion of hilar lesions (b), and age (c) between the training set and the validation set (*P* > 0.05).

**Figure 5:** MRI LAVA dynamic enhanced scanning showed clear hilar features. A 72-year-old female patient presented with hilar infiltrating cholangiocarcinoma. The patient had good breath-holding coordination, clear images at all stages, and no noticeable respiratory artifacts. Plain scan showed irregular thickening of the bile duct wall (a), MRCP image showed significant dilation of the intrahepatic bile duct (b), and images of LAVA dynamic enhancement showed irregular thickening of the hilar bile duct wall with “progressive enhancement” (c–h, arrow).

**Figure 6:** MRI LAVA dynamic enhanced scanning showed unclear hilar features. A 53-year-old female patient with hilar cholangitis had poor breath-holding coordination, and some phase images were not clearly displayed due to the presence of respiratory artifacts. Scan and T2WI coronary (a and b), no obvious abnormal changes; LAVA dynamic enhanced early periods image quality display fair, no obvious respiratory motion artifact (c–h); hepatic portal vein in the bile duct wall thickening of mild change, late to enhance image has the obvious respiratory motion artifact, hepatic portal vein display is not clear, cannot be used for diagnosis.

**Table 1:** The respiratory and pulse scores of patients with hilar lesions in two set.

Group	n	Respiration (times/min)	Pulse (times/min)
Training set	63	18.56 ± 1.37	76.89 ± 6.12
Verification set	27	19.53 ± 1.59	81.42 ± 6.95
*t* value		2.932	3.089
*P* value		0.004	0.003

**Table 2:** Image quality score of patients with hilar lesions in two sets.

Phase	Training set (*n* = 63)					Verification set (*n* = 27)					*P* value
	1	2	3	4	5	1	2	3	4	5	
A1	61	2	0	0	0	18	8	1	0	0	<0.001
A2	58	5	0	0	0	20	5	2	0	0	0.026
A3	60	3	0	0	0	19	7	1	0	0	0.004
A4	40	22	1	0	0	17	7	2	0	1	0.193
A5	37	19	5	0	2	18	5	2	0	2	0.588
A6	32	20	7	1	3	12	9	2	2	2	0.629

## Data Availability

The data used to support the findings of this study are available from the corresponding author upon request.
